This article has been retracted.

# Pimecrolimus Cream 1% in the Management of Atopic Dermatitis in Pediatric Patients: A Meta-Analysis

**DOI:** 10.1371/journal.pone.0093095

**Published:** 2014-04-01

**Authors:** Chunyun Huang, Youyu Sheng

**Affiliations:** Department of Dermatology, Huashan Hospital, Shanghai Medical College, Fudan University, Shanghai, China; University Hospital Hamburg-Eppendorf, Germany

## Abstract

**Objective:**

To evaluate the efficacy and safety of pimecrolimus cream 1% in the treatment of AD in the pediatric population.

**Methods:**

PubMed, EMBASE, Web of Science and Cochrane library databases were searched till July 2013. The randomized and nonrandomized blinded studies of pimecrolimus cream 1% applied twice daily with Jaded score ≥3 in pediatric patients with AD were included. The efficacy outcomes included investigator global assessment (IGA), eczema area and severity index (EASI) scores, pruritus and care giver's assessments and flares free period. Adverse events were reviewed to assess the safety.

**Results:**

Out of 81 studies, 7 were selected that enrolled 2,170 pediatric patients. The pooled analysis reported that pimecrolimus was no better to vehicle reducing eczema at day-8, day-26 and six weeks (OR 4.95, 95% CI 2.79–8.80), (OR 9.69, 95% CI 4.12–22.83) and (OR 3.83. 95% CI 1.94–7.56), respectively in children. Similarly, pimecrolimus did not show beneficial effects when analyzed for mild or absent pruritus at day 4 (OR 8.29, 95% CI 3.88–17.72 favoring vehicle), day 43 (OR 1.81 95% CI 1.13–2.89 favoring vehicle) and 1 week (OR 2.29, 95%CI 1.45 to 3.60 favoring vehicle) as compared with vehicle. One study comparing pimecrolimus with tacrolimus found no significant difference in achieving mild or absent pruritus (OR 0.94, 95% CI 0.44–1.99). More patients showed an improvement in overall disease in vehicle group at day 8 (OR 3.30, 95% CI 2.03–5.35), day 29 (OR 14.14, 95% CI 6.87–29.13) and day 43 (OR 4.11, 95% CI 2.59–6.52) as compared with pimecrolimus 1% group, as assessed by caregivers. No significant difference was seen between the total AEs in both groups (pimecrolimus vs vehicle/tacrolimus) (OR 1.19, 95% CI 0.85, 1.65)

**Conclusion:**

The results of the present meta-analysis showed that pimecrolimus cream 1% was not significantly better to vehicle for AD in pediatrics population.

## Introduction

Atopic dermatitis (AD) also known as atopic eczema, is an inflammatory, chronic and relapsing skin disorder [1] affecting 10% to 15% of the children worldwide [2]. The AD signs and symptoms are seen during first six months of life in 48% to 75% patients [3], [4] and in 80%–85% of the patients at age of five years [5], [6]. There is no consistent overall trend for the incidence or prevalence of atopic eczema worldwide. However, a marked increase in lifetime prevalence of atopic eczema symptoms was seen in Africa, eastern Asia, Western Europe and parts of northern Europe [7].

AD is considered as the first symptom of the ‘atopic march’ [8] and is characterized by itching, redness and skin creases [9]. It has a significant social, personal, emotional and economic impact on the life of patients and their family [10]. Pimecrolimus cream 1% is a promising FDA approved therapy for the clinical care of AD patients [11], [12]. Pimecrolimus cream 1% is an anti-inflammatory compound that blocks the T-cells proliferation and inhibits the production and release of numerous inflammatory mediators from mast cells [12], [13]. It has a unique skin-selective pharmacologic profile [14], [15]. The various clinical trials in infants, children and adults have shown pimecrolimus to be effective in reducing incidence of major flares of the disease; thereby, improving the signs and symptoms of AD [16]–[22]. The treatment of AD with pimecrolimus cream 1% is an important alternative to topical corticosteroids without the associated adverse events (AE) [23], [24].

AD starts in an early age (onset <2 years of age) [9] and is a threat to the overall health and development of a child [25]. The management of AD in children is a complex clinical challenge [10], [26]. Previous studies with pimecrolimus cream 1% have shown it to effective and well tolerated treatment for individuals of all age groups, at all levels of disease severity, irrespective of ethnic origin [11], [17], [27]. It has also been observed to safe and effective on sensitive skin areas such as face and neck [1], [17]. The long term studies have shown that pimecrolimus 1% also improves the quality of life of patients [28].

Pimecrolimus was introduced into the market for the short-term treatment and long term control of AD. It had proved to be effective and safe and tried to replace weaker topical steroids in treatment of AD, however its place in the market is still unclear [13], [29].

Moreover, the clinical data from population of different age groups (infants, children or adults) produces heterogeneity in the results [24]. Little research has been focused on infants [9].The data on long term use of pimecrolimus for AD in children is lacking, as majority of the trials are conducted on population of small sample size. Hence, based on published randomized controlled trials (RCTs) and non-RCTs, we performed a meta-analysis to compare the efficacy and safety of pimecrolimus cream 1% with vehicle or tacrolimus in treating AD specifically in pediatric population.

## Materials and Methods

### Search strategy

A bibliographic search of medical literature till July 2013 was performed using databases as PubMed, EMBASE and Web of Science. The search string (“Pimecrolimus” OR “SDZ ASM 981” OR “ELIDEL”) AND (“atopic dermatitis” OR “dermatitis in children” OR “eczema”) was used to search for relevant articles. The Cochrane library (www.cochranelibrary.com) was also searched. Reference lists of included studies and review articles were manually searched. Only original papers in English published in journals with a peer review process were included after reading the abstracts. The meta-analysis was limited to studies conducted in human.

#### Inclusion and Exclusion Criteria

Blinded, randomized or non-randomized, vehicle controlled or active comparator trials of pimecrolimus cream 1% reporting clinical relevant outcome measures like efficacy, safety or tolerability were selected. The study was eligible for inclusion if 1) the study was on pediatric patients (up to 17 years of age) with diagnosis of AD (mild, moderate or severe); 2) compared topical pimecrolimus 1% with vehicle (cream base, but not containing pimecrolimus) or an active comparator; 3) outcome measures was investigators' global assessment (IGA), eczema area and severity index (EASI), time to first flare or pruritus assessment and; 4) had Jaded score ≥3 [30]. The study was excluded if 1) it was on adult population; 2) an open-labeled study; 3) non-comparative design; 4) either IGA or EASI scores missing; 5) contained previously published data.

The abstract of an article was reviewed if the title of the article and/or key words were relevant. The full text articles of all potentially relevant articles were read to consider the article for inclusion in the study. The reference lists of the included articles were cross checked to identify citations that could have been missed in the primary search steps. The articles reporting insufficient data, using non-standardized scoring systems, or lacking precise comparison methods were rejected. Two authors independently assessed the methodological quality of the included study and extracted the relevant data.

### Intervention

Pimecrolimus cream 1% or corresponding vehicle/active comparator was applied as a thin film to the affected areas twice daily.

### Outcomes

The primary outcome was IGA. EASI was reviewed in the articles wherever available. IGA scores utilize a six-point scale, ranging from 0 (clear) to 5 (very severe disease). IGA scores measure disease severity based on morphology, without referring back to the baseline state [31]. EASI is a validated tool for objectively assessing the severity of eczema. It assesses erythema, infiltration/papulation, excoriation and lichenification separately on a 4-point-scale (0-3), in the head and neck region, trunk, upper limbs and lower limbs [32]. The other efficacy outcome measures were puritus, caregiver assessments and flare free periods.

Adverse events (AEs) were assessed to compare safety. We also compared tolerability profile of pimercrolimus 1% and vehicle by performing a meta-analysis of total withdrawals from each group, discontinuations due to unsatisfactory therapeutic effects and total AEs.

### Data extraction

The meta-analysis was reported as per the Quality of Reporting of Meta-analyses (QUOROM) statement [33]. Two investigators independently assessed the quality of trials and any disagreement was resolved through discussion with the third author. The Jadad score was used to evaluate the quality analysis of methodology, including randomization, blinding and withdrawal from study. The Jadad scale scores from 1 to 5, where 1 or 2 indicates poor in quality and 3–5 indicates high quality [30].

### Statistical analysis

The statistical analysis was performed using software Review Manager 5.2. The output of the data is in the form of forest plot. The population varied in studies that we have selected for example the age of the subject varied from one study to another. Hence, effect size also varied, *i.e*, there was distribution of effect size, so we have used random effect model rather than fixed effect model. We have also investigated heterogeneity by splitting the studies into subgroups and looking at the forest plot and also calculated chi^2^ value. A p-value of <0.1 was considered to be suggestive of statistical heterogeneity. The comparison of the effects between two groups is expressed in terms of odds ratio (OR) and its 95% confidence interval (95% CI). In order to avoid risk of bias, we have included only the blinded, controlled trials and excluded observational and follow up studies.

## Results

### Trial Flow

A total of 81 relative studies published till July 2013 was obtained by electronic databases searches. Of these, 60 were excluded on the basis of title and abstract. The full texts of 21 articles were retrieved and read by two independent investigators. From these 21 articles identified, 14 articles were rejected because of data redundancy, the research goal/objective being different, extension study, an open labeled study, etc. Finally, seven articles (6 randomized and 1 non-randomized) met all entry criteria and were included in the meta-analysis. The trial flow is illustrated in Figure 1.

**Figure 1:** Flowchart of trials.

### Descriptions of studies

The characteristics of the included studies are given in table 1. Of the seven studies, six studies were double-blinded and one was investigator blinded study. A total of 2,170 pediatric patients were enrolled in the included studies. Of these, three trials were conducted on infants (3 to 23 months, n = 638) [19], [20], [34], one on infants and children (3 months to 11 years, n = 275) [35] and three on children and adolescents (2 years to 17 years, n = 1,257) [18], [22]. The severity of participant's AD varied from mild to severe (IGA score = 2 to 4) in five trials [18], [20], [22], [34], [35], mild to moderate (IGA score = 2 to 3) in one trial [19] and moderate to severe (IGA = 3 to 4) in another trial [36].

**Table 1:** Pimecrolimus (Study Characteristics).

Study	Type	n	Age	Center	Severity of AD	Intervention, control	Duration	Outcome
Kapp, 2002	Double-blind, randomized vehicle-controlled parallel-group	251	3–23 months	Multicenter, 41 centers in 8 countries (Belgium, Canada, France, Germany, New Zealand, South Africa, Spain, and the United Kingdom)	Mild to severe	1% pimecrolimus, Vehicle, twice daily	1 year	IGA, EASI, Pruritus
Siegfried, 2006	Double-blind, randomized Vehicle-controlled, parallel-group	275	3 months to 11 years	Multicenter, 35 centers in the United States	Mild to severe	1% pimecrolimus, vehicle, twice daily	6 months	IGA, EASI, Pruritus
Ho, 2003	Double-blind, Vehicle-controlled	186	3–23 months	25 centers in Australia, Brazil, Canada, Germany, South Africa, Spain	Mild to moderate	1% pimecrolimus, vehicle, twice daily	26 weeks **(Double Blind:6 weeks)**	IGA, EASI, Pruritus
Kaufman, 2004	Double blind, randomizedVehicle-controlled	201	3–23 months	Multicenter, 19 centers in Germany	Mild to severe	1% pimecrolimus, Vehicle, twice daily	20 weeks **(Double Blind-4 weeks)**	IGA, EASI, Pruritus, sleep
Wahn, 2002	Double- Blind, randomized vehicle-controlled	713	2–17 years	53 centers in 13 countries (9 in Europe, the United States, Canada, South Africa and Australia	Mild to severe	1% pimecrolimus, Vehicle (Short term treatment: corticosteroids), twice daily	1 year	IGA, EASI
Eichenfiel, 2002	Double-blinded, vehicle controlled, randomized	403	1–17 years	Multicenter	Mild to severe	1% pimecrolimus,twice daily	6 weeks	IGA, EASI
Kemper, 2004	Blinded randomizedParallel-group study	141	2–17 years	Multicenter,19 centers	Moderate to severe	1% pimecrolimus, tacrolimus	26weeks (**6 weeks blinded study)**	IGA

**Vehicle controlled trials.** Six trials (2,029 participants) compared 1% pimecrolimus cream applied twice daily against a vehicle control [18]–[20], [22], [34], [35].

**Active controlled trials.** One trial (141 participants) compared 1% pimecrolimus cream against tacrolimus applied daily [36].

### Efficacy

The efficacy results of different comparisons have been summarized in different figures given below. The efficacy results include IGA, EASI score, flare free periods, improvement in puritus and caregiver assessments. The EASI score of the studies is presented in table 2. Each individual study reported a significantly better reduction (p≤0.0001) in EASI score with pimecrolimus 1% as compared with vehicle.

**Table 2:** Reduction in EASI scores.

Study	Treatment	Vehicle/tacrolimus	Day	P value
Siegfried, 2006	−34%	3%	8	<0.001
Ho, 2003	−81.69%	−25%	43	<0.001
Kaufman, 2004	−71.50	19.4	29	<0.001
Eichenfield, 2002	−45%	1%	43	≤0.001

#### Investigator-rated clinical response as clear or almost clear eczema (reduction in IGA)

The IGA reduction was more with pimecrolimus 1% as compared with vehicle in individual studies. However, when we pooled the data of these individual studies, the reduction in IGA was in favor of vehicle as compared with pimecrolimus 1% at all time points (Figure 2).

**Figure 2:** Analysis of reduction in IGA (Pimecrolimus vs vehicle).

A single trial that compared pimecrolimus 1% with tacrolimus 0.03% (125 participants) found no significant difference between the two groups (OR 0.67 95% CI 0.32–1.40) [36] (Figure 3).

**Figure 3:** Analysis of reduction in IGA (pimecrolimus vs tacrolimus).

#### No flare of eczema during treatment (Flare free periods)

Figure 4 shows the proportion and OR of participants who did not experience a flare of eczema. Kaufmann et al (195 participants) reported significantly more participants without flares in the pimecrolimus group compared against vehicle (OR 0.13, 95% CI 0.05–0.33) within eight days of the treatment [34]. However, at 6 months pimecrolimus did not seem to be beneficial (OR 1.69, 95% CI 1.45 to 1.96 in favor of vehicle) based on data from 3 trials involving 949 participants [20], [22], [35].

**Figure 4:** Analysis of flare free periods (pimecrolimus vs vehicle).

### Mild or absent pruritus

The results of mild or absent pruritus at day 4 (OR 8.29, 95% CI 3.88–17.72), day 43 (OR 1.81 95% CI 1.13–2.89) and 1 week (OR 2.29, 95% CI 1.45 to 3.60) favored vehicle as compared against pimecrolimus. (Figure 5).When compared to tacrolimus, [36] no significant difference was observed in achieving mild or absent pruritus (OR 0.94, 95% CI 0.44–1.99) between the two treatment groups (Figure 6).

**Figure 5:** Analysis of pruritus (pimecrolimus vs vehicle).

**Figure 6:** Analysis of pruritus (pimecrolimus vs tacrolimus).

### Caregiver's assessments

According to care givers assessments, pimecrolimus did not rate better at showing improvement in overall disease (OR 3.30, 95% CI 2.03–5.35 favoring vehicle), day 29 (OR 14.14, 95% CI 6.87–29.13 favoring vehicle) and day 43 (OR 4.11, 95% CI 2.59–6.52 favoring vehicle) as compared with the vehicle group, based on pooled results (Figure 7).

**Figure 7:** Analysis of care giver's assessment (pimecrolimus vs pruritus).

### Adverse Events

The most common adverse events (AEs) were typical childhood infections and ailments. The pooled data for overall AEs showed that there was no significant difference between the total AEs in both groups (OR 1.19, 95% CI 0.85, 1.65) (Figure 8). However, overall study withdrawal (OR 0.44, 95% CI 0.35, 0.55) (Figure 9) and study withdrawal due to unsatisfactory therapeutic effect (OR 0.25, 95% CI 0.19, 0.34) were lesser in pimecrolimus group as compared with vehicle (Figure 10).

**Figure 8:** Analysis of total Adverse events.

**Figure 9:** Analysis of Study withdrawals.

**Figure 10:** Analysis of Study withdrawals due to unsatisfactory therapeutic effects.

## Discussion

The present meta-analysis was conducted to compare pimecrolimus 1% to vehicle/active comparator for the treatment of pediatrics AD. Seven double-blinded/investigator blinded, randomized/non-randomized, vehicle controlled/active comparator, multicentre studies were identified and the data was pooled and analyzed. We compared IGA, EASI score, pruritus assessments, care givers assessments and flare free periods of these studies. The safety of pimecrolimus cream 1% vs. vehicle and active comparator was also assessed in children. Overall, the results of this meta-analysis showed that pimecrolimus cream 1% was not significantly better to vehicle for AD in children.

AD is common disease of children with an overall prevalence of 10-15-%, [2], however, little data is available to assess its management in children. Pimecrolimus is a non-steroid inhibitor of inflammatory cytokines [14] and is thought to be an important treatment for children as it does not induce skin atrophy [37]. Majority of the clinical trials with pimecrolimus have been carried out in adults and have shown promising results [21], [38]–[40].

Evidence from short-term studies (4 weeks to 6 weeks) has shown that topical pimecrolimus 1% is safe and effective for the treatment of AD in infants [19], [34], [35] while the long term studies (6 to 12 months) have shown that pimecrolimus 1% significantly reduces the incidence of disease flares; thereby, controlling the signs and symptoms of AD [20], [22]. In the present meta-analysis, the three studies on very young population (3 to 23 months of age) have reported substantial clinical benefits in terms of safety and tolerability of pimecrolimus 1%. While the two studies on children and adolescents concluded that the use of pimecrolimus 1% to treat early signs and symptoms prevented the progression of major AD flares. However, the pooled results of these studies in meta-analysis did not yield promising results for pimecrolimus.

Ashcroft et al conducted a meta-analysis of 25 RCTs on 4186 patients using pimecrolimus 1% or tacrolimus 0.1% or 0.03% Both the drugs were significantly more effective than a vehicle control. However, the review was unable to show the long term safety of pimecrolimus or tacrolimus over corticosteroids. Also, due to absence of key comparisons with tacrolimus, the clinical importance for topical pimecrolimus was unclear [24]. In our meta-analysis, we were able to identify only one study that compared pimecrolimus 1% with tacrolimus 0.03% in pediatric patients. The study showed that though both had similar efficacy, but pimecrolimus achieved better tolerability than tacrolimus. However, it is difficult to comments on the efficacy of pimecrolimus as compared with tacrolimus through the data of a single study.

Chen et al in a meta-analysis of 20 trials involving 6288 infants and children with AD reported that both the treatments are safe and effective in pediatric patients with AD, with tacrolimus being superior to pimecrolimus. However, the authors have reported the possibility of evaluation bias of remissive effects in this systematic review [31].

A Cochrane review from 31 clinical trials, involving 8019 participants observed that treatment of AD with pimecrolimus was effective when compared against vehicle. Again, this systematic review did not find evidence to support that pimecrolimus was better option to treat eczema than moderate or potent corticosteroids or tacrolimus. The pooled results reported no statistically significant difference between 1.0% pimecrolimus and 0.03% tacrolimus in achieving clear or almost clear of eczema and mild or absent pruritus following 1 week of the treatment [28].

We comprehensively searched for blinded, controlled trials from a wide range of databases in order to avoid the risk of publication bias, and used clinically relevant outcome measures. However, our meta-analysis has certain limitations. Due to a lack of relevant comparative data the clinical role of pimecrolimus is uncertain. Further, there is little evidence to support the use of pimecrolimus in infants. We compared rates of withdrawals, unsatisfactory therapeutic effects, and total AEs that were based on data pooled from trials of different durations. Moreover, long term safety (beyond 1 or 2 years) of use of pimecrolimus is lacking because it has been in use for less than a decade. Hence, long term trials are required in future to check its long term efficacy.

Though the present meta-analysis from large number of patients from more than 192 centers gives a doubtful view in the use of pimecrolimus 1% in infants and children, we suggest that pimecrolimus should be used with caution in this population taking in to consideration the clinical condition of these patients and available management strategies for AD in children.

## Supporting Information

Checklist S1 **PRISMA Checklist.**
(DOCX)

## References

[1] HebertAA (2006) Review of pimecrolimus cream 1% for the treatment of mild to moderate atopic dermatitis. Clinical therapeutics 28: 1972–1982.1729645410.1016/j.clinthera.2006.12.014

[2] Schultz LarsenF (1993) The epidemiology of atopic dermatitis. Monographs in allergy 31: 9–28.8450851

[3] KayJ, GawkrodgerDJ, MortimerMJ, JaronAG (1994) The prevalence of childhood atopic eczema in a general population. Journal of the American Academy of Dermatology 30: 35–39.827702810.1016/s0190-9622(94)70004-4

[4] Wadonda-KabondoN, SterneJA, GoldingJ, KennedyCT, ArcherCB, et al (2003) A prospective study of the prevalence and incidence of atopic dermatitis in children aged 0–42 months. The British journal of dermatology 149: 1023–1028.1463280910.1111/j.1365-2133.2003.05605.x

[5] EmersonRM, WilliamsHC, AllenBR (2001) What is the cost of atopic dermatitis in preschool children? The British journal of dermatology 144: 514–522.1126000810.1046/j.1365-2133.2001.04077.x

[6] Hywel C, Williams, David P, Strachan (1997) The Challenge of Dermato-Epidemiology. CRC Press Inc.

[7] DeckersIA, McLeanS, LinssenS, MommersM, van SchayckCP, et al (2012) Investigating international time trends in the incidence and prevalence of atopic eczema 1990–2010: a systematic review of epidemiological studies. PloS one 7: e39803.2280806310.1371/journal.pone.0039803PMC3394782

[8] XuF, YanS, LiF, CaiM, ChaiW, et al (2012) Prevalence of childhood atopic dermatitis: an urban and rural community-based study in Shanghai, China. PloS one 7: e36174.2256348110.1371/journal.pone.0036174PMC3341360

[9] HoareC, Li Wan PoA, WilliamsH (2000) Systematic review of treatments for atopic eczema. Health technology assessment 4: 1–191.PMC478281311134919

[10] SuJC, KempAS, VarigosGA, NolanTM (1997) Atopic eczema: its impact on the family and financial cost. Archives of disease in childhood 76: 159–162.906831010.1136/adc.76.2.159PMC1717083

[11] EichenfieldLF, LuckyAW, LangleyRG, LyndeC, KaufmannR, et al (2005) Use of pimecrolimus cream 1% (Elidel) in the treatment of atopic dermatitis in infants and children: the effects of ethnic origin and baseline disease severity on treatment outcome. International journal of dermatology 44: 70–75.1566366710.1111/j.1365-4632.2004.02234.x

[12] GuptaAK, ChowM (2003) Pimecrolimus: a review. Journal of the European Academy of Dermatology and Venereology: JEADV 17: 493–503.1294108110.1046/j.1468-3083.2003.00692.x

[13] Graham-BrownRA, GrassbergerM (2003) Pimecrolimus: a review of pre-clinical and clinical data. International journal of clinical practice 57: 319–327.12800465

[14] StuetzA, GrassbergerM, MeingassnerJG (2001) Pimecrolimus (Elidel, SDZ ASM 981)- preclinical pharmacologic profile and skin selectivity. Seminars in cutaneous medicine and surgery 20: 233–241.1177091010.1053/sder.2001.29066

[15] GrassbergerM, SteinhoffM, SchneiderD, LugerTA (2004) Pimecrolimus — an anti-inflammatory drug targeting the skin. Experimental dermatology 13: 721–730.1556075510.1111/j.0906-6705.2004.00269.x

[16] StaabD, KaufmannR, BrautigamM, WahnU (2005) Treatment of infants with atopic eczema with pimecrolimus cream 1% improves parents' quality of life: a multicenter, randomized trial. Pediatric allergy and immunology: official publication of the European Society of Pediatric Allergy and Immunology 16: 527–533.1617640110.1111/j.1399-3038.2005.00306.x

[17] WellingtonK, NobleS (2004) Pimecrolimus: a review of its use in atopic dermatitis. American journal of clinical dermatology 5: 479–495.1566334510.2165/00128071-200405060-00013

[18] EichenfieldLF, LuckyAW, BoguniewiczM, LangleyRG, CherillR, et al (2002) Safety and efficacy of pimecrolimus (ASM 981) cream 1% in the treatment of mild and moderate atopic dermatitis in children and adolescents. Journal of the American Academy of Dermatology 46: 495–504.1190749710.1067/mjd.2002.122187

[19] HoVC, GuptaA, KaufmannR, ToddG, VanaclochaF, et al (2003) Safety and efficacy of nonsteroid pimecrolimus cream 1% in the treatment of atopic dermatitis in infants. The Journal of pediatrics 142: 155–162.1258453710.1067/mpd.2003.65

[20] KappA, PappK, BinghamA, Folster-HolstR, OrtonneJP, et al (2002) Long-term management of atopic dermatitis in infants with topical pimecrolimus, a nonsteroid anti-inflammatory drug. The Journal of allergy and clinical immunology 110: 277–284.1217026910.1067/mai.2002.126500

[21] MeurerM, Folster-HolstR, WozelG, WeidingerG, JungerM, et al (2002) Pimecrolimus cream in the long-term management of atopic dermatitis in adults: a six-month study. Dermatology 205: 271–277.1239967610.1159/000065863

[22] WahnU, BosJD, GoodfieldM, CaputoR, PappK, et al (2002) Efficacy and safety of pimecrolimus cream in the long-term management of atopic dermatitis in children. Pediatrics 110: e2.1209398310.1542/peds.110.1.e2

[23] BreuerK, BraeutigamM, KappA, WerfelT (2004) Influence of pimecrolimus cream 1% on different morphological signs of eczema in infants with atopic dermatitis. Dermatology 209: 314–320.1553989510.1159/000080855

[24] AshcroftDM, DimmockP, GarsideR, SteinK, WilliamsHC (2005) Efficacy and tolerability of topical pimecrolimus and tacrolimus in the treatment of atopic dermatitis: meta-analysis of randomised controlled trials. BMJ 330: 516.1573112110.1136/bmj.38376.439653.D3PMC552812

[25] KrakowskiAC, EichenfieldLF, DohilMA (2008) Management of atopic dermatitis in the pediatric population. Pediatrics 122: 812–824.1882980610.1542/peds.2007-2232

[26] AkdisCA, AkdisM, BieberT, Bindslev-JensenC, BoguniewiczM, et al (2006) Diagnosis and treatment of atopic dermatitis in children and adults: European Academy of Allergology and Clinical Immunology/American Academy of Allergy, Asthma and Immunology/PRACTALL Consensus Report. Allergy 61: 969–987.1686705210.1111/j.1398-9995.2006.01153.x

[27] PappKA, WerfelT, Folster-HolstR, OrtonneJP, PotterPC, et al (2005) Long-term control of atopic dermatitis with pimecrolimus cream 1% in infants and young children: a two-year study. Journal of the American Academy of Dermatology 52: 240–246.1569246810.1016/j.jaad.2004.09.016

[28] Ashcroft DM, Chen LC, Garside R, Stein K, Williams HC (2007) Topical pimecrolimus for eczema. The Cochrane database of systematic reviews: CD005500.10.1002/14651858.CD005500.pub2PMC1004387117943859

[29] WilliamsH (2002) New treatments for atopic dermatitis. BMJ 324: 1533–1534.1208907310.1136/bmj.324.7353.1533PMC1123485

[30] JadadAR, MooreRA, CarrollD, JenkinsonC, ReynoldsDJ, et al (1996) Assessing the quality of reports of randomized clinical trials: is blinding necessary? Controlled clinical trials 17: 1–12.872179710.1016/0197-2456(95)00134-4

[31] ChenSL, YanJ, WangFS (2010) Two topical calcineurin inhibitors for the treatment of atopic dermatitis in pediatric patients: a meta-analysis of randomized clinical trials. The Journal of dermatological treatment 21: 144–156.2039449010.3109/09546630903401470

[32] HanifinJM, ThurstonM, OmotoM, CherillR, TofteSJ, et al (2001) The eczema area and severity index (EASI): assessment of reliability in atopic dermatitis. EASI Evaluator Group. Experimental dermatology 10: 11–18.1116857510.1034/j.1600-0625.2001.100102.x

[33] MoherD, CookDJ, EastwoodS, OlkinI, RennieD, et al (1999) Improving the quality of reports of meta-analyses of randomised controlled trials: the QUOROM statement. Quality of Reporting of Meta-analyses. Lancet 354: 1896–1900.1058474210.1016/s0140-6736(99)04149-5

[34] KaufmannR, Folster-HolstR, HogerP, ThaciD, LofflerH, et al (2004) Onset of action of pimecrolimus cream 1% in the treatment of atopic eczema in infants. The Journal of allergy and clinical immunology 114: 1183–1188.1553642910.1016/j.jaci.2004.08.015

[35] SiegfriedE, KormanN, MolinaC, KianifardF, AbramsK (2006) Safety and efficacy of early intervention with pimecrolimus cream 1% combined with corticosteroids for major flares in infants and children with atopic dermatitis. The Journal of dermatological treatment 17: 143–150.1685475310.1080/09546630600647297

[36] KempersS, BoguniewiczM, CarterE, JarrattM, PariserD, et al (2004) A randomized investigator-blinded study comparing pimecrolimus cream 1% with tacrolimus ointment 0.03% in the treatment of pediatric patients with moderate atopic dermatitis. Journal of the American Academy of Dermatology 51: 515–525.1538918510.1016/j.jaad.2004.01.051

[37] Queille-RousselC, PaulC, DuteilL, LefebvreMC, RapatzG, et al (2001) The new topical ascomycin derivative SDZ ASM 981 does not induce skin atrophy when applied to normal skin for 4 weeks: a randomized, double-blind controlled study. The British journal of dermatology 144: 507–513.1126000710.1046/j.1365-2133.2001.04076.x

[38] GollnickH, KaufmannR, StoughD, HeikkilaH, AndrianoK, et al (2008) Pimecrolimus cream 1% in the long-term management of adult atopic dermatitis: prevention of flare progression. A randomized controlled trial. The British journal of dermatology 158: 1083–1093.1834166510.1111/j.1365-2133.2008.08484.x

[39] LugerTA, LahfaM, Folster-HolstR, GulliverWP, AllenR, et al (2004) Long-term safety and tolerability of pimecrolimus cream 1% and topical corticosteroids in adults with moderate to severe atopic dermatitis. The Journal of dermatological treatment 15: 169–178.1520415010.1080/09546630410033781

[40] MeurerM, FartaschM, AlbrechtG, VogtT, WormM, et al (2004) Long-term efficacy and safety of pimecrolimus cream 1% in adults with moderate atopic dermatitis. Dermatology 208: 365–372.1517892810.1159/000078462

